This article has been retracted.

# Pseudopyronine B: A Potent Antimicrobial and Anticancer Molecule Isolated from a *Pseudomonas mosselii*

**DOI:** 10.3389/fmicb.2016.01307

**Published:** 2016-08-26

**Authors:** S. Nishanth Kumar, S. R. Aravind, Jubi Jacob, Geethu Gopinath, Ravi S. Lankalapalli, T.T. Sreelekha, B.S. Dileep Kumar

**Affiliations:** ^1^Agroprocessing and Natural Products Division, National Institute for Interdisciplinary Science and Technology – Council of Scientific and Industrial ResearchThiruvananthapuram, India; ^2^Laboratory of Biopharmaceuticals and Nanomedicine, Division of Cancer Research, Regional Cancer CentreThiruvananthapuram, India

**Keywords:** *Pseudomonas mosselii*, Pseudopyronine B, antimicrobial, anticancer activity, apoptosis

## Abstract

In continuation of our search for new bioactive compounds from soil microbes, a fluorescent *Pseudomonas* strain isolated from paddy field soil of Kuttanad, Kerala, India was screened for the production of bioactive secondary metabolites. This strain was identified as *Pseudomonas mosselii* through 16S rDNA gene sequencing followed by BLAST analysis and the bioactive metabolites produced were purified by column chromatography (silica gel) and a pure bioactive secondary metabolite was isolated. This bioactive compound was identified as Pseudopyronine B by NMR and HR-ESI-MS. Pseudopyronine B recorded significant antimicrobial activity especially against Gram-positive bacteria and agriculturally important fungi. MTT assay was used for finding cell proliferation inhibition, and Pseudopyronine B recorded significant antitumor activity against non-small cell lung cancer cell (A549), and mouse melanoma cell (B16F10). The preliminary MTT assay results revealed that Pseudopyronine B recorded both dose- and time-dependent inhibition of the growth of test cancer cell lines. Pseudopyronine B induced apoptotic cell death in cancer cells as evidenced by Acridine orange/ethidium bromide and Hoechst staining, and this was further confirmed by flow cytometry analysis using Annexin V. Cell cycle analysis also supports apoptosis by inducing G_2_/M accumulation in both A549 and B16F10 cells. Pseudopyronine B treated cells recorded significant up-regulation of caspase 3 activity. Moreover, this compound recorded immunomodulatory activity by enhancing the proliferation of lymphocytes. The production of Pseudopyronine B by *P. mosselii* and its anticancer activity in A549 and B16F10 cell lines is reported here for the first time. The present study has a substantial influence on the information of Pseudopyronine B from *P. mosselii* as potential sources of novel drug molecule for the pharmaceutical companies, especially as potent antimicrobial and anticancer agent.

## Introduction

The discovery of antibiotics has decreased the spread and severity of a broad range of infectious diseases caused by human pathogenic microbes. However, due to the wide spread use of antibiotics, the competence of many introduced antibiotics in the market is being threatened by the rise of microbial pathogens which are resistance to the current clinical chemotherapeutic agents (Cowan, 1999). Human infections owing to multi-drug-resistant microbes is a serious challenge to many patients, especially those, are in hospitals (Arias and Murray, 2009; Fischbach and Walsh, 2009). Infectious diseases account for more than 13 billion human deaths worldwide, which accounts for about 25% of all deaths (Zin et al., 2011). The antibiotic treatments of various infectious diseases are also getting limited due to the reemergence of multi-drug-resistance (MDR) pathogenic microbes, which have been frequently reported from many parts of the world. Methicillin-resistant *Staphylococcus aureus* (MRSA) is one of the important drug resistant pathogen, which is frequently reported by many clinicians worldwide. A part from MRSA and VRSA (vancomycin resistant *S. aureus*), several other drug resistant and pan-drug-resistant (PDR) microbes especially Gram-negative bacteria, including carbapenem resistant *Pseudomonas aeruginosa, Enterococcus faecium, Klebsiella pneumoniae, Acinetobacter baumannii, Enterobacter* sp*.*, and *Stenotrophomonas maltophilia*, are emerging as an important health problem to human being (Huang et al., 2013). Recently, few novel drugs have been industrialized exactly for treating various Gram-negative MDR/PDR bacteria (Payne et al., 2006; Vaara et al., 2010; Velkov et al., 2010). Many bioactive compounds from natural sources have played an important role in the discovery of many antibiotics which are used clinically. Moreover, 70% of the clinically used antimicrobials are either unchanged natural compounds used directly or derived from natural compounds by synthetic tailoring (Singh et al., 2011). Thus, more investigation should be initiated for discovering and developing novel antimicrobial molecules especially from natural sources is urgently needed.

At present, one in four deaths in the USA is because of various tumors (Fadeyi et al., 2013). When classified within age groups, the tumor is one of the five important reasons of death among humans (males and females) and the single major cause of human death around the world (Fadeyi et al., 2013). By 2016, cancer morbidity may increase more than 10 million worldwide. This growing tendency also indicates a shortage in the various current tumor treatments including surgical operation, chemotherapy, and radiotherapy. Since the normal endurance rates of cancer have remained essentially unaffected in spite of such above mentioned hostile treatments, so there is an urgent requirement for new anticancer drugs with advanced efficiency, and fewer side effects that can be developed at a reasonable price to common people worldwide.

Tawiah et al. (2012) reported that “Throughout the various years, natural compounds are the most constantly fruitful basis of diverge bioactive metabolites having several applications in the field of modern human medicine, pharmaceutics and agriculture.” Therefore, the search for new antimicrobials from natural sources is an important area of many researchers worldwide. Microorganisms from soils play an important source of many novel antibiotic compounds due to their high abundance and amazing diversity. There are many reports of the production of antimicrobial metabolites by *Pseudomonas* spp. Some of these antimicrobials have been chemically characterized, and their commercial exploitation is attempted (Zhou et al., 2012).

As mentioned earlier infectious diseases and cancer is the most leading cause of death worldwide. Therefore, novel and potent therapeutic agents are often required to control these diseases. To achieve this goal, several new sources of antimicrobial/anticancer compounds ranging from natural to synthetic are currently being explored worldwide. Therefore in our continuous search for new bioactive secondary metabolites from soil bacteria, Pseudopyronine B was purified from a *Pseudomonas mosselii* TR strain. The current manuscript also reported the antimicrobial and anticancer activity of Pseudopyronine B.

## Materials and Methods

### Chemicals and Media Used in Current Study

All the chemicals and reagents used in the current study were of the finest purity. All the chemicals used for separation and purification of bioactive compounds were from Merck (Mumbai, India). Silica gel (mesh size: 230–400) used for column purification and precoated silica gel 60 plates (GF_254_) used for thin layer chromatography (TLC) were purchased from Merck (Germany). Various media used for microbiological investigation were purchased from Hi-Media Laboratories Pvt. Ltd, Mumbai, India. The antibiotics ciprofloxacin and amphotericin B, which were used as standard positive control, were procured from Sigma-Aldrich (USA). The Chemsketch Ultra (Toronto, ON, Canada) software was used for drawing the chemical structure.

### Bioactive Compound Producing Bacterium

A fluorescent *Pseudomonas*, named as TR strain was isolated from paddy field of Kuttanad region of Kerala, India was used in the present study. Kuttanad is a unique agroclimatic zone in India where paddy is cultivated below sea level and is blessed with a rich microbial population which is not fully explored for economic cultivation. The strain was identified as a fluorescent *Pseudomonas* strain through classical identification methods.

### Molecular Identification of TR Strain through 16S rDNA Sequencing

#### Extraction of Bacterial DNA and Sequencing of the 16S Gene

A pure culture of bacteria was raised in 10 ml of Luria-Bertani broth (LB) for 18 h to obtain OD value of approximately 0.7 at 600 nm. The bacterial culture broth (1.5 ml) was pelleted in a microfuge tube for 2 min at 12,000 rpm. Total DNA was extracted using standard phenol–chloroform extraction procedures (Sambrook et al., 2001). PCR amplification was done with universal primers (f: 5′-GATTAGATACCCTGGTAGTCCAC-3′ and r: 5′-CCCGGGAACGTATTCACCG-3′) specific for the 16S rDNA gene. The PCR reaction was carried out in a total volume of 50 μl [DNA (100 ng), MgCl_2_ (4 Mm), PCR reaction buffer (1X, Genei, Bangalore, India), each deoxyribonucleotide triphosphate (2.5 mM), Taq polymerase (1.5 U, Genei, Bangalore, India) and each primer (40 pmol)]. PCR cycle conditions were: 2 min initial denaturation at 95°C, followed by 36 cycles of denaturation for 30 s at 95°C, followed by 1 min primer annealing at 60°C and 1 min primer extension at 72°C. Final primer extension step was carried for 2 min at 72°C. PCR amplification was achieved on a Bio-Rad Thermal Cycler (USA). Amplicons were analyzed in 1% (w/v) agarose gels. The gels were stained with an aqueous solution containing ethidium bromide (0.5 mg/mL) and visualized on a UV transilluminator. Amplicons were purified using the QIA quick purification kit (Qiagen, Valencia, CA, USA) and sequenced. The sequencing was performed on an ABI PRISM 310 Genetic analyzer (Perkin-Elmer Applied Biosystems, Foster City, CA, USA) using the universal primers (described for PCR amplification) and the Big Dye Terminator Cycle Sequencing Ready Reaction Kit (Perkin-Elmer, Applied Biosystems). The 16S rDNA gene sequences (partial) obtained were finally aligned using ABI Prism software (Perkin-Elmer, Applied Biosystems) and compared to sequences retrieved from GenBank Database and BLAST.

#### Phylogenetic Analysis

The phylogenetic investigation was performed using MEGA 6.0 software program (Molecular Evolutionary Genetics Analysis, Version 6.0; Tamura et al., 2007). The phylogenetic tree topologies were assessed by bootstrap analyses based on 1000 replicates, and final phylogenetic trees were constructed with the neighbor-joining method as reported earlier (Saitou and Nei, 1987). The taxonomic position of the present strain was recognized based on 16S rDNA homology.

#### Fermentation and Extraction of Crude Bioactive Secondary Metabolites

The bacterial production and solvent extraction of crude bioactive secondary metabolites from TR strain were done according to George et al. (2015) in King’s B media (KB). The supernatant was collected according to the method of George et al. (2015) and extracted with ethyl acetate trice (1:1 v/v) in a globe shaped separating funnel (2 L) and the ethyl acetate portion was collected, concentrated and dried in a Buchi rota evaporator (40°C) for further detailed investigations.

#### Purification of Bioactive Compound

Activated silica gel (230–400 mesh) was filled into a 600 mm × 30 mm long glass column using n-hexane solvent. The crude secondary metabolite (0.85 g) was subjected to silica gel column chromatography purification, with a elution profile of 5% ethyl acetate (EtOAc), 10% EtOAc, 20% EtOAc, 40% EtOAc in hexane (100 ml each), 50% EtOAc in hexane (150 ml), 100% EtOAc (100 ml), 5% MeOH in EtOAc (100 ml), obtained 75 fractions. The purity of the fractions was determined by TLC. An aliquot of each collected fraction was spotted on the activated TLC plates (silica gel 60; 10 cm × 10 cm). Ethyl acetate and hexane (1:1) was used for developing TLC plates. Spots were positioned by UV and further revealing the TLC plate to iodine vapors. One fraction (tubes 35–37) was obtained as pure. This fraction was evaporated to give a faint white residue (17 mg). Initial bioactivity of this fraction was confirmed by testing against *Bacillus subtilis*, which was used as indicator test microorganism.

#### Identification of the Bioactive Compound

The NMR spectra (^1^H NMR and ^13^C) of the pure compound were documented using a Bruker DRX500 NMR spectrometer (Bruker, Rheinstetten, Germany) at room temperature and the chemical shifts are reported relative to the corresponding reference solvent (methanol). HR-ESI-MS of the compound was recorded using a Thermo Scientific Exactive Mass Spectrometer (Thermo Fisher 110 Scientific, USA) with an electrospray ionization mode.

### Antimicrobial Activity of the Compound

#### Pathogenic Microbes Used in the Study

##### Bacterial

The following Gram-positive and negative pathogenic bacteria are used for antibacterial study. Gram-positive pathogenic bacteria: *B. subtilis* (MTCC 2756), *Bacillus cereus* (MTCC 430), *S. aureus* (MTCC 902), *S. epidermis* (MTCC 435), and *S. simulans* (MTCC 3610); Gram-negative pathogenic bacteria: *Escherichia coli* (MTCC 2622), *Klebsiella pneumoniae* (MTCC 109), *Proteus mirabilis* (MTCC 425), *Proteus vulgaris* (MTCC 1771), *P. aeruginosa* (MTCC 2642), *Salmonella typhi* (MTCC 3216), and *Vibrio cholerae* (MTCC 3905).

##### Fungal

The fungal strains used in the present are *Aspergillus flavus* (MTCC 183), *A. fumigatus* (MTCC 3376), *A. niger* (MTCC 282), *A. tubingensis* (MTCC 2425), *Colletotrichum gloeosporioides* (MTCC 2151), *Fusarium oxysporum* (MTCC 284), *Penicillium expansum* (MTCC 2006), *Rhizoctonia solani* (MTCC 4634), and *Trichophyton rubrum* (MTCC 296).

All the test microbes were obtained from MTCC (Microbial Type Culture Collection and GenBank), Council of Scientific and Industrial Research- Institute of Microbial Technology (CSIR-IMTECH), Chandigarh, India.

### Determining the Antibacterial Activity of Test Compound

#### Minimum Inhibitory Concentration (MIC) and Minimum Bactericidal Concentration (MBC)

The MIC of the compound was determined according to broth microdilution method as suggested by Clinical and Laboratory Standard Institute, USA (Clinical and Laboratory Standards Institute [CLSI], 2012a). Briefly, the concentration of the fresh overnight culture of test bacteria was adjusted to 1 × 10^5^ CFU/ml using a spectrophotometer. Dilutions of inocula were cultured on a Nutrient agar (NA) medium to check the validity of the inoculum and the absence of any contaminations. Different solvent and water dilutions of test compound (0.5–1000 μg/ml) and ciprofloxacin (0.25–250 μg/ml) were placed in the wells containing 150 μl of nutrient broth (NB), followed by the addition of 10 μl of inoculum. After that, the ELISA plates were incubated for 18–24 h at 37°C. After incubation MIC was determined by measuring the OD at 600 nm. The lowest concentration of test compound that produced a significant inhibition (around 90%) of the growth of the bacteria in comparison with the positive control was identified as the MIC.

About 100 μl from the ELISA wells not displaying any microbial growth in the MIC test were diluted serially using 0.85% saline and plated on NA plates to determine the MBC values. The NA plates were incubated at 37°C for 24 h. MBC is defined as the lowest concentration of antibacterial agent that reduces the viability of the initial bacterial inoculum by 99.99%.

#### Disk Diffusion Experiment of Test Compound

The antimicrobial activity of the pure compound was performed by the disk diffusion assay against the test bacterial pathogens as mentioned by CLSI, USA (Clinical and Laboratory Standards Institute [CLSI], 2012b). The test bacterial strain preserved in NA at 4°C were sub-cultured in NB to get the working concentration approximately containing 1 × 10^6^ CFU/ml. The test compound (MIC concentration) was loaded into a sterile disk (Hi-Media) with 6 mm diameter. Then Mueller-Hinton agar (MHA) plates were swabbed with each test bacterial pathogens and the compound loaded disks were placed along with the control antibiotics disk. Here, ciprofloxacin disks (5 μg/disk) were used as the standard positive control and the plates were incubated for 24 h at 37°C until bacteria had developed in a confluent film. The antimicrobial property of the test compound and antibiotic was determined by measuring the zone of inhibition (diameter) expressed in mm. The experiment was performed in triplicate sets.

### Determining the Antifungal Activity of Test Compound

#### Minimum Inhibitory Concentration

The MIC of test compound against the fungi was done by broth microdilution assay as per the recommendations of Clinical and Laboratory Standard Institute, USA (Clinical and Laboratory Standards Institute [CLSI], 2010, 2012c), with RPMI 1640 growth medium supplemented by L-glutamine, without sodium bicarbonate (all from Sigma-Aldrich) and buffered to pH 7.0 according to the previously reported method (Aravind et al., 2014). The lowest concentration of agents that produced a significant inhibition (90%) of the growth of the test fungi in comparison with the standard positive control was defined as the MIC.

#### Disk Diffusion Experiment of Test Compound

The compound was screened for their antifungal activity against test fungi by agar disk diffusion experiment as mentioned by CLSI, USA (Clinical and Laboratory Standards Institute [CLSI], 2008, 2009). Briefly, PDA plates were inoculated (0.1 ml) with a spore suspension in 0.85% sterile saline. The concentration of test fungal suspension was adjusted to 1 × 10^5^ CFU/ml using sterile saline. The test compound (MIC concentrations) was loaded into a 6-mm diameter sterile filter paper disks (Hi-Media, India), air dried and then placed on the surface of the PDA plates swabbed previously by test fungi. The plates were incubated at 35°C for 48–72 h. After incubation, the antifungal activity was assessed by measuring the zone of inhibition (diameter) and expressed in millimeter (mm). The assay was performed in triplicate sets.

### Anticancer Studies of the Test Compound

#### Cancer Cell Lines Used in the Study: Its Source and Maintenance and Treatments

The following three cancer cell lines were used in the present investigation (1) Non-small cell lung cancer (A549), (2) mouse melanoma cell (B16F10) and (3) liver cancer cell (HepG2) lines and these cell lines were obtained from NCCS (National Centre for Cell Science), Pune, India and maintained throughout the study in Dulbecco’s Modified Eagle Medium (DMEM) added with 3 mM of L-glutamine, 100 μg/ml of streptomycin, 100 IU/ml of penicillin, 10% heat inactivated (56°C) fetal bovine serum (FBS) and 25 mM of HEPES [4-(2-hydroxyethyl)-1-piperazineethanesulfonic acid]. The final pH was adjusted to 7.2 by bicarbonate solution at 37°C in a CO_2_ incubator.

Stock solutions (3 mg/500 μl) of the test compound, made in dimethyl sulfoxide (DMSO), were further dissolved in the corresponding medium (DMEM) to the necessary working concentrations. A549, B16F10 and HepG2 cell lines were seeded into ELISA plates and incubated for 24 h at 37°C in a CO_2_ incubator. After the cell adherence, six different concentrations of test compound (0.1, 1, 5, 10, 50, and 100 μg/ml) were added to the wells containing test cancer cell lines, except to the control wells. Control wells contain only DMEM nutrient medium and the test cells. The cultures were incubated for various time periods (24, 48, and 72 h).

#### Anti-proliferative Activity

The cytotoxic effect of the test compound was determined by MTT [3-(4,5-dimethylthiazol-2-yl)-2,5-diphenyltetrazolium bromide] methods as described earlier (Aravind et al., 2015). The concentrations used in this study are 0.1, 1, 5, 10, 50, and 100 μg/ml.

### Apoptosis Induction Assay Using the Test Compound

#### Acridine Orange and Ethidium Bromide Staining (AO/EB Staining)

Apoptotic morphology of cancer cells after treatment with Pseudopyronine B was investigated by staining the cancer cells with a combination of the fluorescent DNA-binding acridine orange (AO) and ethidium bromide (EB) dyes to decide the viable and non-viable cancer cells in a population. Cells were collected and washed three times with PBS after being incubated with IC_50_ concentration of Pseudopyronine B for 24, 48 and 72 h, and were then stained with 100 μg/ml AO/EB stain (Sigma-Aldrich) for 2 min. Then the color and structure of the cancer cells were immediately recorded under an inverted fluorescence microscope (Aravind et al., 2014).

#### Detection of Morphological Apoptosis with Hoechst 33342 Staining

The morphological apoptosis like chromatin condensation in the test cancer cell lines was observed by nuclear staining dye Hoechst 33342 (Aravind et al., 2014). After treatment with Pseudopyronine B (IC_50_ concentration) for 24, 48 and 72 h, the A549 and B16F10 cells were washed with PBS trice and then further fixed with methanol: acetic acid (3:1) for 10 min at room temperature in the dark. Fixed cells were again washed with PBS and stained with 1 μg/ml of Hoechst 33342 stain (10 mg/ml) for 10 min in the dark at room temperature. Changes in the nuclei of cells after staining with Hoechst 33342 were recorded using an inverted fluorescence microscope (stimulation at 350 nm and emission at 460 nm; Leica, Germany).

#### Annexin V/Propidium Iodide Assay

The annexin V/propidium iodide (PI) method was done according to the recommendation given by manufacturer’s (Invitrogen, USA). Briefly, A549 and B16F10 cell lines were seeded into six well plates and incubated for 24, 48, and 72 h with Pseudopyronine B (IC_50_ concentration). After incubation, the cells were collected and washed with ice-cold PBS and centrifuged. The pellet was resuspended in 100 μl of binding buffer containing 2.5 μl FITC conjugated Annexin V and 1 μl 100 μl/ml PI and incubated for further 15 min at room temperature in the dark. A total of at least 10000 events were composed and examined by BD flow cytometry (BD Biosciences, San Jose, CA, USA; Liu et al., 2013).

#### Cell Cycle Analysis of Cancer Cells after Treatment with Test Compound

The cellular DNA content and distribution in the cell cycle were enumerated by BD flow cytometry using PI staining. A549 and B16F10 cells were seeded in the T_25_ culture flask and treated with Pseudopyronine B (IC_50_ concentration) for the various time periods (24, 48, and 72 h). Cells were collected, washed with PBS twice, and fixed in 70% ethanol at -20°C. After fixation, the cells were washed in PBS and centrifuged. The pellets thus obtained was treated with RNase (1 mg/ml; Roche, Mannheim, Germany) at 37°C for 30 min and then incubated with PI for at least 30 min. Cell-cycle analysis was recorded with the FACS Calibur Flow Cytometer (BD Biosciences, San Jose, CA, USA) and the data were analyzed with Flowjo software.

#### Determination of Activation of Caspase 3

Caspase-Glo assay kits (Promega) were used to determine the activation of Caspase 3 by following manufacturer’s instructions. A549 and B16F10 cells were plated into ELISA plates and incubated for 24 h. After 24 h seeding, cells were treated with test compound (5, 10, and 50 μg/ml) and incubated for 48 h. Subsequently, 100 ml of caspase-3 assay reagent was added to each well. After adding the reagent, the plate was incubated for 1 h in the dark and the luminescence was quantified with the help of a microplate reader (SpectraMax M5, Molecular Devices). The activity of Caspase was expressed as a percentage (%) of the untreated control treatment (DMSO). The experiment was performed in triplicate (Wang et al., 2014).

#### Proliferation Assay of Normal Lymphocytes

The proliferation of normal lymphocytes when treated with test compound was done as described earlier (Aravind et al., 2014).

### Statistical Analysis

Disk diffusion data was presented as mean ± standard deviation. The error bars represent ± SD. taken from three independent experiments. Statistical analysis was performed with SPSS (Version 17.0; SPSS, Inc., Chicago, IL, USA). The significance level was set at *P* < 0.05.

## Results

### Based on 16S rDNA Sequencing and Phylogenetic Analysis, Bacteria Was Identified as *P. mosselii*

Molecular characterization of the TR bacterium (*P. mosselii*) was performed by 16S rDNA gene sequencing. PCR amplification of 16S rDNA gene yielded -1500 bp amplicon. BLAST analysis recorded 99% similarity to *P. mosselii* 16S rDNA sequence accessible in the NCBI GenBank database and based on this our TR strain was identified as *P. mosselii*. The partial 16S rDNA gene sequence data have been deposited in the NCBI GenBank nucleotide database under the accession number KF712283. The phylogenetic tree clearly portrayed the relationships our *P. mosselii* with other *Pseudomonas* strains used for the present analysis. The present TR bacterial isolate (*P. mosselii* strain) was very successfully clustered along with other *P. mosselii* sequences obtained from the NCBI GenBank database further confirming the authenticity of our isolate (**Figure 1**). The *P. mosselii* was currently deposited in CSIR-IMTECH (Institute of Microbial Technology, Chandigarh, India).

**FIGURE 1:** **Phylogenic tree displaying the relationships of *Pseudomonas mosselii* TR strain and other known *Pseudomonas* species based on 16S rDNA gene sequences (Neighbor-joining Method)**.

### The Bioactive Compound Was Identified as Pseudopyronine B Based on Detailed Spectral Analyses

Ethyl acetate fraction of *P. mosselii* yielded one main compound, which having an R_f_ value 0.68. Initial bioactivity of this compound was confirmed by testing the antimicrobial activity against *B. subtilis* and the compound recorded significant activity (data not shown). The compound was identified based on the spectral data as Pseudopyronine B (**Figure 2**).

**FIGURE 2:** **(A)** Structure of Pseudopyronine B and **(B)** HR–MS spectra of Pseudopyronine B.

Pseudopyronine B:^1^H NMR (500 MHz, CD_3_OD) δ 0.91 (2 × t, *J* = 6.8 Hz, 2 × 3 H), 1.27–1.39 (m, 14 H), 1.42–1.50 (m, 2 H), 1.66 (quin, *J* = 7.3 Hz, 2 H), 2.38 (t, *J* = 7.5 Hz, 2 H), 2.48 (t, *J* = 7.5 Hz, 2 H), 5.99 (s, 1 H); ^13^C NMR (126 MHz, CD_3_OD) δ 12.9, 13.0, 22.2, 22.3, 22.4, 26.5, 27.5, 28.5, 28.6, 28.8, 29.2, 31.4, 31.5, 32.9, 99.6, 102.5, 163.7, 166.4, 167.4; ESI-MS [M+H]^+^ C_18_H_31_O_3_ calc′d for m/z 295.22732, found 295.22729.

### Antibacterial Activity of Pseudopyronine B

The Pseudopyronine B was tested for checking its antibacterial (MIC and MBC) activity against 13 bacterial species using standard CLSI protocol and the values are presented in **Table 1**. Pseudopyronine B recorded significant antibacterial activity against Gram positive bacteria, while most of the tested Gram negative bacteria recorded no activity. The microorganism that presented highest sensitivity toward Pseudopyronine B was *S. epidermis* (1 μg/ml), followed by *S. aureus* (4 μg/ml). The diameter of zone of inhibition obtained from agar disk diffusion experiment was presented in **Table 1** and *S. epidermis* recorded significant diameter of zone of inhibition (33 mm) and is shown in **Figure 3**. The activity of Pseudopyronine B against *S. epidermis* was superior to ciprofloxacin, standard antimicrobial agent (**Table 1**).

**Table 1:** Antibacterial activity of Pseudopyronine B.

Test bacteria	Pseudopyronine B			Ciprofloxacin		
		
	MIC (μg/ml)	MBC (μg/ml)	Zone of inhibition (Diagram in mm)	MIC (μg/ml)	MIC (μg/ml)	Zone of inhibition (Diagram in mm)
*B. subtilis*	64	125	20 ± 1	2	2	30 ± 1
*B. cereus*	16	32	23 ± 0	1	2	31 ± 1.52
*S. aureus*	4	4	31 ± 0.23	1	2	33 ± 1.14
*S. epidermis*	1	2	33 ± 0.56	2	4	30 ± 1.77
*S. simulans*	8	8	28 ± 1.72	4	4	29 ± 0.56
*E. coli*	–	–	–	1	2	27 ± 0.77
*P. mirabilis*	–	–	–	0.5	1	29 ± 0.56
*P. vulgaris MTCC 1771*	–	–	–	2	4	30 ± 1.15
*V. cholerae*	–	–	–	2	4	31 ± 1.72
*K. pneumonia*	4	8	25	1	2	25 ± 1.15
*P. aeruginosa*	–	–	–	2	4	27 ± 0
*S. typhi*	32	32	22	4	4	29 ± 1


*–, recorded no activity.*

**FIGURE 3:** **Antimicrobial activity of Pseudopyronine B**.

### Antifungal Activity of Pseudopyronine B

Antifungal property of Pseudopyronine B against 11 fungi and the MIC values are shown in **Table 2**. Pseudopyronine B documented good antifungal property especially against plant pathogenic fungi. Pseudopyronine B displayed best MIC value against *P. expansum* (4 μg/ml), followed by *F. oxysporum* and *R. solani* (16 μg/ml). In agar disk diffusion assay *P. expansum* recorded significant activity (34 mm; **Table 2**; **Figure 3**).

**Table 2:** Antifungal activity of Pseudopyronine B.

Test bacteria	Pseudopyronine B		Amphotericin B	
		
	MIC (μg/ml)	Zone of inhibition (Diagram in mm)	MIC (μg/ml)	Zone of inhibition (Diagram in mm)
*A. flavus*	16	21 ± 0.52	4	23 ± 1.15
*A. fumigatus*	64	18 ± 0.77	2	27 ± 1.72
*A. niger*	32	21 ± 1.12	2	26 ± 0.56
*A. tubingensis*	–	–	4	30 ± 0.77
*C. gloeosporioides*	–	–	32	25 ± 1.12
*F. oxysporum*	16	25 ± 1.12	125	26 ± 2.21
*P. expansum*	4	34 ± 0.52	64	23 ± 2.27
*R. solani*	16	24 ± 1	64	23 ± 072
*T. rubrum*	–	–	2	24 ± 0.56


*–, recorded no activity.*

### Anticancer Activity

#### Pseudopyronine B Recorded Significant Anti-proliferative Activity as Evidenced by MTT Assay

Anti-proliferative activity of Pseudopyronine B was assessed on non-small cell lung cancer (A549), mouse melanoma cell (B16F10) and liver cancer cell (HepG2) lines. MTT assay was used to evaluate the cell viability after Pseudopyronine B treatment. From the MTT experiment it is clearly evident that the Pseudopyronine B recorded both dose- and time-dependent inhibition in the growth of test cancer cell lines, when treated with 100, 50, 10, 5, 1, and 0.5 μg/ml (**Figure 4A**). Out of three cell lines tested, A549 and B16F10 cells recorded best activity. A549 and B16F10 cells turned out to be the most sensitive cell lines and were selected for further apoptotic studies.

**FIGURE 4:** **(A)** Cytotoxicity profile of Pseudopyronine B on A549 and B16F10 cells measured by MTT assay. **(B)** Phase contract images of A549 and B16F10 cells treated with Pseudopyronine B. The experiments where performed in three replication and results were expressed as mean ± standard deviation.

### Apoptotic Induction Assays

#### Pseudopyronine B Induces Apoptosis in A549 and B16F10 as Evidenced by Acridine Orange-Ethidium Bromide and Hoechst 33342 Staining

The cultured A549 and B16F10 cells were examined for their morphology features after treatment with Pseudopyronine B. It was observed that the Pseudopyronine B is inducing characteristic apoptosis features changes such as nuclear condensation, membrane blebbing and formation of apoptotic bodies, when compared to untreated control as evaluated by phase contrast microscope. Moreover, there was a significant reduction in the number of A549 and B16F10 cells after Pseudopyronine B treatment (**Figure 4B**). Acridine orange-ethidium bromide staining was done to confirm the nuclear membrane damage, a characteristic feature of apoptosis as observed by yellow/orange coloration in the nuclei of A549 and B16F10 cells treated with Pseudopyronine B (**Figure 5**). The cells treated with the compound after 24, 48 and 72 h exhibited time depend increase in AO-EB positivity, when compared to untreated control (**Figure 5**).

**FIGURE 5:** **Analysis of A549 and B16F10 cell lines to detect apoptosis by Acridine orange/ethidium bromide staining.** In this method live cells were detected as green color, whereas the apoptosis cells documented orange-red due to the co-staining of acridine orange with ethidium bromide stain due to the loss of membrane integrity by the action of Pseudopyronine B.

The Hoechst 33342 staining of A549 and B16F10 cells recorded a very significant increase in the number of cancer cells showing nuclear condensation and fragmentation after treatment with Pseudopyronine B when examined through phase contrast microscope (**Figure 6**). Moreover, cancer cells lost its normal structure after treatment with Pseudopyronine B and presented an expansion of the endoplasmic reticulum. Some very specific signs of early stages of apoptosis (vacuolization in the cytoplasm, nucleus shrinkage and fragmentation and chromatin densification) can also be viewed in Pseudopyronine B treated cells through phase contrast microscope (**Figure 6**).

**FIGURE 6:** **Hoechst staining of A549 and B16F10 cells.** Treatment with Pseudopyronine B resulted in apoptotic death.

#### Effect of Pseudopyronine B on Cell Cycle Analysis

Distribution of cells on the different phases of the cell cycle was investigated by flow cytometry after treatment of A549 and B16F10 cells with several concentrations of Pseudopyronine B for 24, 48, and 72 h. In both A549 and B16F10 Pseudopyronine B treated cells, G1 and G2/M phase were increased were as S phases found to be decreased. In A549 cells at 48 h of incubation control cells possess 68.96 ± 2.94% in G1 phase were as in Pseudopyronine B treated cells have 76.36 ± 2.67%. Control cells in G2/M phase possess 5.88 ± 0.84% were as in Pseudopyronine B treated cells have 11.88 ± 1.04%. In B16F10 cells at 48 h of incubation control cells possess 70.62 ± 3.56% and 72.79 ± 3.21% for Pseudopyronine B treated cells. In G2/M phase control cells possess 17.59 ± 1.59% and 21.12 ± 1.64% for Pseudopyronine B treated cells suggesting that it can induce significant apoptosis in A549 and B16F10 cells (**Figure 7**).

**FIGURE 7:** **Effect of Pseudopyronine B against A549 and B16F10 on cell cycle.** The experiments where performed in three replication and results in bar diagram were expressed as mean ± standard deviation.

#### Pseudopyronine B Induces Apoptotic Events by Altering Membrane Permeability as Evidenced by Flow Cytometry

Annexin V-FITC staining, using flow cytometry was used to detect the morphological changes that occur in the early stages of apoptotic cells (**Figure 8**). After 48 h of treatment, Pseudopyronine B induced apoptosis on A549 [14.1 ± 1.34% in control to 76.5 ± 2.97% in Pseudopyronine B treated cells (*P* < 0.001)] and B16F10 [21.7 ± 1.68% in control to 64.7 ± 2.67% in Pseudopyronine B treated cells (*P* < 0.001)] cells.

**FIGURE 8:** **Pseudopyronine B induce phosphatidylserine exposure in A549 and B16F10 cells.** The cells were stained with annexin V-FITC and propidium iodide. Analyses were performed by flow cytometry. Each data represents mean ± SD from three independent experiments.

#### Pseudopyronine B Induces Caspase 3 Activation in Cells

Our next attempt was to examine the basic mechanism behind the cytotoxic effect of Pseudopyronine B. For this, we tested the activation of caspase 3 using a colorimetric assay. Pseudopyronine B treated cells and control lysates were prepared and incubated with Ac-DEVD-pNA caspase 3 specific substrate with the reaction buffer and the caspase 3 pNA release was measured using a spectrophotometer at 405 nm. Significant enhancement in the caspase 3 activity was recorded in Pseudopyronine B treated cells when compared with that of control clearly indicating the involvement of caspase 3 in Pseudopyronine B induced apoptotic cell death (**Figure 9**). The results are given in **Figure 9**.

**FIGURE 9:** **Effect of Pseudopyronine B on the release of caspase 3 in A549 and B16F10 cells.** The experiments where performed in three replication and results were expressed as mean ± standard deviation.

#### Evaluation of Immunomodulatory Properties of Pseudopyronine B

Immunomodulatory activity of Pseudopyronine B was checked by the proliferation of lymphocyte. The proliferation lymphocyte was slightly enhanced in Pseudopyronine B treated cells when compared to that of control cells (untreated). The proliferation index of lymphocyte was detected to be 1.08 for 5 μg/ml of Pseudopyronine B in the presence of PHA (**Figure 10**).

**FIGURE 10:** ***In vitro* lymphocyte proliferative activity of Pseudopyronine B after 72 h of incubation period**.

## Discussion

The enormous rise in the value of drug discovery and development is a strong encouragement for many pharmaceutical industries to contempt all but the most economically bioactive lead molecules (Higginbotham et al., 2013). But, the decreasing quantity of medicines reaching the market is putting strong pressure on the pharmaceutical companies to research and find alternative sources for novel lead molecules (Bennani, 2012). Natural molecules with diverse bioactivity have been used since the beginning of various conventional medicines in early years (Graca et al., 2013). These bioactive molecules are present in all forms of life and are usually produced during the secondary metabolism by almost all organisms. A wide variety of structurally interesting and bioactive secondary metabolites produced by various microorganisms including bacteria, fungi, actinomycetes, etc. have been reported worldwide and many of them are taken by the several pharmaceutical companies as lead drug molecules especially antibiotics (Gao et al., 2012). Several microbes especially from terrestrial soils have an inborn capability of producing many novel natural molecules with various biological properties and this represent rich source of biologically active compounds which may play very important role in drug discovery process for pharma industry (Bode et al., 2002). In the present study, a bacterial strain, named as TR, was isolated from soil during a screening for microbes with potent antimicrobial property. The microbial strain used in the present study was identified as a *P. mosselii* strain based 16 S rDNA sequencing and BLAST analyses.

There are many literature reports on the production of compounds with antimicrobial properties by *Pseudomonas* spp. Some of these antimicrobial compounds have been identified chemically and the structure has been reported (Zhou et al., 2012). Several fluorescent *Pseudomonas* spp. have currently received world-wide interest due to the production of a board range of bioactive compounds with antibiotics properties such as phenazine-1-carboxylic acid, pyoluteorin, phenazine-1-carboxamide, viscosinamide and tesin (Chin-A-Woeng et al., 2003; Hu et al., 2005; Huang et al., 2009) and several bioactive enzymes. In this study, *P. mosselii* exhibit remarkable antimicrobial property especially against a broad range of plant pathogenic fungi, Gram-positive and negative human pathogenic bacteria. So far, many antibiotics have been isolated and identified from *Pseudomonas* species, and most of them were from *P. aeruginosa*, which is the most studied species of *Pseudomonas*. *P. mosselii* is one of the *Pseudomonas* species that has not been studied extensively. In the present study we have isolated Pseudopyronines B from *P. mosselii* and the isolation of Pseudopyronine B from *P*. *mosselii* is reported here for the first time.

The isolation of Pseudopyronines A and B is previously reported from marine sponge associated *Pseudomonas* species collected from the Fiji islands (Singh et al., 2003, 2011; Kong et al., 2005) and *Pseudomonas* sp. associated with entomopathogenic nematode (Grundmann et al., 2012). These compounds showed significant MICs against Gram-positive bacteria, including *S. aureus, B. subtilis*, methicillin-resistant *S. aureus* and *Enterococcus faecium* (MIC value: 2–4 μg/ml) and reasonable activity against *E. faecalis* and *S. pneumoniae* (MIC value: 16–64 μg/ml) with being the more active of the two compounds (Giddens et al., 2008; Singh et al., 2011). Similar results were observed in our study also (**Table 1**), where in our study also *Staphylococcus* spp. recorded best activity. Antimycobacterial activity of pseudopyronines against *M. tuberculosis* H37Rv is also well-reported in the literature (Giddens et al., 2008). Pseudopyronines are powerful and comparatively selective parasitic protozoa (*Leishmania donovani*) inhibitors (Blunt et al., 2010). These reports clearly portrait the role of Pseudopyronines in modern drug discovery process. The antifungal activity of Pseudopyronines especially Pseudopyronine B is not reported in literature. In the present manuscript the antifungal activity of Pseudopyronine B especially against plant pathogenic fungi is reported for the first time.

Bioactive compounds especially from natural have played a significant role over several years in the growth of various anticancer drugs. Many natural compounds and their derivatives have been successfully categorized according to the standard collection of several cancer drugs, such as paclitaxel, vinblastine, and vincristine (Zhong et al., 2012). Newman et al. (2003) reported that more than 50% of the novel compounds approved between 1982 and 2002 were derived directly or indirectly from natural compounds. This clearly indicated that natural compound play a profound role in the development of various anticancer drugs. Even though cancer is the leading cause of mortality worldwide and most of the chemotherapeutic compounds already in clinic have been reported to exhibit severe toxicity to normal cells, accompanied by other unwanted side effects to our body. Moreover, most of these compound are highly expensive, mutagenic, and carcinogenic (Cao et al., 2010). Therefore, it is very important to find out low toxic anti-cancer agents from natural sources. In this study, Pseudopyronine B was isolated from natural source and was tested for its cytotoxicity effect on A549, B16F10, and HepG2 cancer cell lines. We showed that Pseudopyronine B effectively inhibited cell growth of A549 and B16F10. When compared to that of A549 and B16F10 cells, Pseudopyronine B treated HepG2 cells recorded less activity. Alterations in the apoptosis and its related signaling pathways have a vital role in the development of tumor (Cao et al., 2010). Pseudopyronine B treated A549a and B16F10 cells exhibited typical morphological features of apoptosis including membrane flip-flop, cell shrinkage, higher uptake of stain with apoptotic markers and finally end up in severe DNA damage. The faults in apoptosis pathway are supposed to be one of the important causes of human cancer (Thompson, 1995). Thus, a compound which induces apoptosis in cancer cells are one of the most efficient approaches in treating cancer (Lowe and Lin, 2000).

The exact mode of action of Pseudopyronine B remains unclear. Using acridine orange-ethidium bromide and Hoechst staining assay, we observed that Pseudopyronine B induced apoptosis and DNA damage in A549 and B16F10 cell lines. Interesting in all most all cases, cellular DNA is the major goal of many chemotherapeutic drug molecules, which directly or indirectly attach to DNA. These drugs also obstruct DNA metabolism and inhibit the action of DNA polymerases and/or topoisomerases, which intern inhibit cell replication. Usually apoptosis occurs, following cellular DNA damage. Cysteine-containing aspartate-specific proteases (caspases) in the cells play a very important role in the activation of various apoptotic signaling pathways. So far, 10 members have been identified in humans. Caspase-8 and caspase-9 are two initiator caspases which are capable of transducing apoptosis signals by direct activation of downstream executioner caspase-3 (Chen et al., 2003). Caspase-3, a protein on the common path of cell apoptosis, is one of the most important members and the key executor of cell apoptosis. Caspase-3 usually exists in the cytoplasm in the form of an inactive zymogen. When activated by the many external apoptosis signals, caspase-3 can induce the inactivation of many key proteases in the cytoplasm, cell nucleus, and cytoskeleton, and finally cause the apoptosis of cells. In the current study, cleavage of caspase-3 and up regulation of its cleaved form in A549 and B16F10 cells treated with Pseudopyronine B revealed Pseudopyronine B-induced apoptosis occurred through the caspase-3-dependent pathway.

Cellular apoptosis (programmed cell death) is a common form of cell death induced by many anticancer compounds/drugs (Vaux and Korsmeyer, 1999). Apoptosis cells are well-categorized by various morphological defects, such as condensation of chromatin, membrane flip-flop, and the formation of apoptotic body. These changes in cancer cells were finally leads to DNA fragmentation which was observed as a ladder on agar gel electrophoresis (Desagher and Martinou, 2000; Nonpunya et al., 2014). Apoptosis is mainly induced by a caspase cascade or translocation of apoptosis inducing factors (Nonpunya et al., 2014). There are two important pathways in the activation of caspase, which are the cell surface death receptor (extrinsic pathway) and mitochondrial initiator (intrinsic pathway). Caspase-3 and caspase-7 is the “execute” caspase for the apoptotic induction, while caspase-8 and caspase-9 are the critical caspases and signify the activation of the extrinsic and intrinsic pathways, respectively (McConkey, 1998; Law et al., 2014). The activation of caspases plays a significant role during apoptotic cell death; especially, the caspase 3 activation and activation of this caspase is an important step in the apoptosis procedure (Elmore, 2007). Interestingly Pseudopyronine B recorded enhanced activation of caspase 3, which may play an important role in apoptosis in A549 and B16F10 cells.

## Conclusion

Here, it is highly evident from the present findings that a *P*. *mosselii* which produces a powerful bioactive substance (Pseudopyronine B), active against bacteria especially Gram-positive. The present study contributes to the quest for novel antimicrobial compounds, a vital strategy in emerging alternative therapies to treat many infections caused by pathogenic microbes. Pseudopyronine B also recorded significant antifungal activity against plant pathogenic fungi. Isolation of Pseudopyronine B from *P*. *mosselii* and antifungal activity is reported here for the first time. Although, the present study delivers some valuable basic information about Pseudopyronine B from *P*. *mosselii* and further detailed investigation are needed to determine their potential for clinical applications.

In the present study, we confirmed that Pseudopyronine B inhibiting cell growth in a dose- and time-dependent manner. We also demonstrated that the cell death is due to apoptosis. To our best knowledge, this is the first investigation reporting the anticancer activity of Pseudopyronine B, which has the potential to be evaluated as a novel anticancer drug. Further studies are warranted to decipher the molecular mechanisms by which Pseudopyronine B modulates programmed cell death in various cancer cells. More over the results in the present study clearly point out the potential therapeutic property of Pseudopyronine B as an anticancer agent.

## Author Contributions

SNK performed experiments, analysis, or interpretation of data and manuscript preparation; SA performed anticancer section; JJ performed purification of compound; GG helped in manuscript preparation; TS performed anticancer section; RL performed purification of compound; BDK designed the work and manuscript correction.

## Conflict of Interest Statement

The authors declare that the research was conducted in the absence of any commercial or financial relationships that could be construed as a potential conflict of interest.
